# The Chronotropic Function of Propofol and the Underlying Mechanism in Rabbits

This article has been retracted.

**DOI:** 10.1155/2021/5222745

**Published:** 2021-11-15

**Authors:** Wenjie Cheng, Xiaohua Sun, Yanfang Liu, Shiqi Han, Wanlu Ren

**Affiliations:** Department of Anesthesiology, Tianjin Hospital, Tianjin 300211, China

## Abstract

The report of bradycardia caused by propofol is increasing. In the experiment, we investigated the chronotropic function of propofol and the underlying mechanism. Rabbits of both sexes were randomly divided into 4 groups: propofol 5 mg/kg group, 10 mg/kg group, 15 mg/kg group, and sham group. Heart rate and frequency of vagal efferent discharge were recorded before the injection and 0, 0.5, 1, 2, and 10 min after the injection through intravenous mode. Then, their hearts were removed, and sinoatrial nodes were dissected. The action potentials of the sinus node pacemaker cells were recorded by the intracellular glass microelectrode technique, and the sinoatrial (SA) node was exposed to propofol 1, 3, 5, and 10 *µ*M respectively. The action potentials were recorded after the sinoatrial nodes were exposed to each concentration of propofol for 15 min. Our results show that the heart rate significantly decreased, and the vagal efferent discharge was significantly increased at 0, 0.5, 1, and 2 min after the injection, respectively. Besides, as the dose increases, the magnitude of change shows a dose-dependent manner. Propofol exerts a negative chronotropic action on sinoatrial node pacemaker cells. The drug significantly decreased APA, VDD, RPF, and prolonged APD_90_ in a concentration-dependent manner. These effects may be the main mechanism of propofol-induced bradycardia in clinical study.

## 1. Introduction

Propofol is a kind of fat-soluble, rapid short-acting intravenous anesthetic, which has the advantages of quick onset, short duration, and quick recovery. It has gradually become the preferred drug for clinical induction and maintenance of anesthesia and has been widely used in various surgical anesthesia and can significantly reduce the occurrence of perioperative adverse events [1, 2]. With the wide application in clinic, the report of bradycardia caused by this drug is increasing [3, 4].

Although propofol-induced bradycardia has been recognized for several years, the pathophysiologic mechanism is not completely understood. It is generally agreed that bradycardia is regulated by the propofol antisympathetic effect. However, some studies showed that the decrease of heart rate induced by propofol could not be completely explained by the effect of the central vagus nerve, that is, propofol may also have a direct inhibitory effect on the sinoatrial (SA) node [5, 6].

In this study, electrocardiogram and neuroelectrophysiological techniques were used to observe the changes of heart rate and discharge frequency of the vagus nerve after intravenous administration of propofol in rabbits. Furthermore, the effect of propofol on the automechanism of isolated rabbit sinoatrial node cells was investigated by the intracellular microelectrode recording technique, to confirm the direct effect of propofol on the sinoatrial node. The results of our experiment provide a theoretical basis for the clinical interpretation of bradycardia caused by propofol.

## 2. Materials and Methods

### 2.1. Protocol I

Animal experiments were approved by the Animal Care and Use Committee of the Hebei Medical University and performed in accordance with the National Institutes of Health guidelines for the Care and Use of Laboratory Animals. Healthy rabbits weighing 1.8–2.2 kg, male and female, were collected and divided into 4 groups (*n* = 6) according to the random number table: propofol 5 mg/kg group (group P1), propofol 10 mg/kg group (group P2), propofol 15 mg/kg group (group P3), and sham group (group C). The experimental group was intravenously injected with different doses of propofol, while the control group received an equal amount of 0.9% saline instead.

The rabbits were anesthetised by intravenous injection of 3% pentobarbital sodium 1 ml/kg along the ear margin. After supine fixation, acupuncture electrodes were inserted into the extremities to detect ECG activity. After that, the muscle tissue was separated through a median incision in the neck, and the carotid artery sheath was exposed along the right side of the trachea. The right vagus nerve trunk was separated with a glass minute hand under an operating microscope, and the peripheral end was pinched. The surrounding nerve was moisturized with a warm paraffin film to prevent nerve dryness and insulate from the surrounding tissue. The vagus nerve was placed on a platinum electrode (2 mm apart) to guide the discharge, and the vagus nerve was immersed in warm paraffin oil. During the experiment, 8 ml/kg of normal saline was added to the auricular vein, and infrared heat was used to keep the anal temperature of the animals at about 37°C.

Acupuncture electrodes were connected with a Caidiofax S multichannel electrocardiogram (ECG-1250C) to monitor ECG activity. The discharge signal of the vagus nerve is connected to AVB-11 bioelectric amplifier (Nihon Kohden, Japan) and then displayed on a VG-10 oscilloscope (Nihon Kohden, Japan). The amplified signal is connected to a BL-420S biological signal acquisition system (Techman, China) and recorded. The duration of recording was 60s, the sampling stenography was 1 kHz/s, and the filtering range was 100∼1000 Hz.

#### 2.1.1. Record of Heart Rate and Vagus Nerve Discharge

Heart rate and discharge frequency of the vagus nerve were recorded at the following time points: before injection (T0), immediately after injection (T1), 0.5 (T2), 1 (T3), 2 (T4), and 10 min (T5) after injection.

### 2.2. Protocol II

#### 2.2.1. Electrophysiological Measurements

After the first part of the experiment, the hearts of rabbits were quickly excised. The region of the right atrium bounded by the crista terminalis and the superior and inferior vena cava, and the interatrial septum were dissected free from the adjacent tissues in Tyrode's solution (−4°C). The preparations were pinned down on a thin silicon disc on the base of a perfusion chamber and equilibrated for 1h. The Tyrode's solution was prepared with deionized, distilled water and composed of (in mmol/L) NaCl, 136.8; KCl, 5.4; CaCl, 21.08; MgCl, 21.25; NaHCO_3_, 1.2; tris, 5.0; and glucose, 11.0. It was oxygenated with 95%O_2_ and 5%CO_2_ and maintained at 36 ± 0.5°C with a pH of 7.40 ± 0.03. The transmembrane potentials were recorded by KCl-filled (3 mol/L) micropipettes with tip diameter less than 0.5 *µ*m, coupled to a high input impedance amplifier (MEZ8201, Nihon Kohden, Japan). The amplified signals were fed to the A/*D* converter and processed by a microcomputer. The amplitude of action potential (APA), rate of pacemaker firing (RPF), APD at 90% repolarization (APD_90_), and velocity of diastolic depolarization in phase 4 (VDD) were recorded.

#### 2.2.2. Electrophysiological Effects of Propofol on SA Node Pacemaker Cells

The experiment started after the preparation was equilibrated for 1h in Tyrode's solution at a perfusion rate of 5 ml/min. The effects of propofol on action potentials (APs) were studied in a cumulative manner. After recording of 3 control Aps, propofol at 1, 3, 5, and 10 *µ*M was applied, and APs were recorded at 15 min after application of each concentration of propofol.

#### 2.2.3. Statistical Analysis

Statistical analysis was performed using SPSS21.0 (SPSS Inc., IL, USA). All data were expressed as mean ± standard deviation (SD). The differences in the parameters between pre- and postapplication of were compared using Student's *t*-test. For multigroup comparison, one-way analysis of variance (ANOVA) with Bonferroni post hoc test was used to determine statistical significance. Statistical significance was considered as *P* < 0.05.

## 3. Results

### 3.1. Effect of Propofol on Heart Rate in Rabbits

In the control group, normal saline was injected intravenously, no significant change of heart rate was observed. However, the heart rate was significantly lower than the baseline value at T1, T2, T3, and T4 time points after propofol injection (*P* < 0.05) and presented concentration-dependence. At T5 time point, the heart rate recovered in each group, compared with T0, and no significant difference was found (*P* > 0.05). The results are shown in Table 1 and Figure 1(a).

### 3.2. Effect of Propofol on the Discharge Frequency of Vagus Nerve in Rabbits

The spontaneous discharge of vagus nerve was not observed in the control group after intravenous injection of normal saline. However, the efferent discharge of the vagus nerve increased significantly than the baseline value at the T1, T2, T3, T4 time point after propofol injection (*P* < 0.05), and showing a concentration dependence. Compared with T0, there was no significant difference in the vagus nerve discharge at 10 min after propofol injection (*P* > 0.05). The results are shown in Table 2 and Figure 1(b).

### 3.3. Electrophysiological Effects of Propofol on SA Node Pacemaker Cells

Compared with the control group, propofol (1, 3, 5 *µ*M) showed concentration-dependent inhibitory effects on the sinus node of rabbits. The experimental results suggest that propofol could reduce the action potential parameters APA, VDD, RPF, and prolong APD_90_. Action potential parameters of pacemaker cells did not change after high concentration of propofol (10 *µ*M) was superfused. The results are shown in Table 3 and Figures 2 and 3.

## 4. Discussion

As a kind of fat-soluble, rapid short-acting intravenous anesthetic, propofol has the advantages of quick onset, short duration, and quick recovery, which is suitable for rapid induction and maintenance in general anesthesia. Besides, the stress response during tracheal intubation could be reduced by propofol during anesthesia induction. In addition, a large number of studies proved that propofol has protective effects against perioperative organ injury [7, 8]. Due to the advantages, propofol is widely used in outpatient, surgical anesthesia, and ICU sedation. With the wide application in clinic, the report of bradycardia caused by this drug is increasing [3].

At present, it is believed that propofol produces sedative or anesthetic effects mainly through the positive regulation of the inhibitory function of neurotransmitter GABA by acting on ligand-gated GABA receptors [9]. Therefore, we hypothesize that central vagal excitation mediates the propofol-induced bradycardia. In our study, the changes of the efferent discharge of the cervical vagus nerve induced by propofol were directly observed by the in vivo electrophysiological method. The results are consistent with our hypothesis that intravenous propofol can increase the efferent discharge frequency of cervical vagus nerve. Previous studies indicated that the load-dose of propofol can dramatically increase the plasma concentration in the body, and the half-life of the drug is 2–4 minutes [10]. Our results suggest that propofol increased discharge of the vagus nerve, leading to a concentration-dependent decrease in heart rate, which is consistent with the above conclusion. Compared with the baseline at T0, there was no difference in the discharge of the vagus nerve at 10 min after intravenous administration, which was considered to be related to propofol pharmacokinetic characteristics.

Previous studies showed that the heart rate decrease induced by propofol could not be fully explained by the central vagus effect, that is, it may also have a direct inhibitory effect on the sinoatrial node [5]. In this study, we observed the effect of propofol on the action potential of pacemaker cells in the isolated rabbit sinoatrial node. The experimental results showed that, in a certain range, propofol had a concentration-dependent inhibitory effect on the sinoatrial node in rabbits, which means the drug had a direct effect of lowering heart rate in the periphery. In addition, this effect did not change after high dose of propofol, indicating that this inhibition may have a capping effect. It was confirmed that the level of maximum repolarization potential, threshold potential, and the speed of 4-phase automatic depolarization affected the automaton of the pacemaker cells in the SA node. The rate of depolarization of the 4-phase depends on the growth rate of the net inward current, which in turn depends on the relative ratio of the internal Ca^2+^ flow and the external K^+^ flow [11]. If some factor promotes Ca^2+^ influx or suppresses K^+^ outflow, the increase of net inward current will be accelerated during 4-phase automatic depolarization, which will lead to the increase of pacing cell automatics. On the contrary, the automaticity is reduced. Based on the results that propofol could concentration-dependently reduce the action potential parameters APA, VDD, RPF, and prolong APD90 in the second part of our experiment, we hypothesized that propofol may reduce the autonomic activity of the pacemaker cells in the rabbit sinus node by inhibiting calcium channels, but the exact mechanism needs to be further investigated.

There are some limitations to this study. First, we did not explore the exact mechanism of the propofol regulation heart rate. The effect of propofol may be involved in other central nerve pathways. Second, considering clinically relevant concentration and referring to a previous study [12, 13], we only choose 5 mg/kg, 10 mg/kg, and 15 mg/kg propofol intravenous, but different doses of propofol were not tested. Third, the exact mechanism by which propofol reduces the automaticity of the sinoatrial node was not investigated. Last, we did not discuss the countermeasures for bradycardia induced by propofol. In view of the experimental results, we believe that low-dose atropine is safe and effective in preventing bradycardia.

## 5. Conclusions

Taken together, these results demonstrate that intravenous administration of propofol and the heart rate of rabbits decreased, and the efferent discharge frequency of cervical vagus nerve increased correspondingly. In addition, propofol has a negative time-varying effect on pacemaker cells of the sinoatrial node in rabbits. The combination of the central and peripheral effects may be the reason for the chronotropic function after intravenous propofol in the clinic.

## Figures and Tables

**Figure 1:** Heart rate and frequency of the vagus nerve between groups. Heart rate and discharge frequency of the vagus nerve were recorded at the following time points: before injection (T0), immediately after injection (T1), 0.5 (T2), 1 (T3), and 2 (T4), and 10 min (T5) after injection. (a) Heart rate. (b) Frequency of vagus nerve. Sham group; P1: 5 mg/kg propofol group; P2: 10 mg/kg propofol group; and P3: 15 mg/kg propofol group. Data are expressed as mean ± SD. ^*∗*^*P* < 0.05 vs. sham; ^#^*P* < 0.05 vs. P1; ^**+**^*P* < 0.05 vs. P2.

**Figure 2:** Electrophysiological effects of propofol on sinoatrial node pacemaker cells. The action potential parameters APA, VDD, RPF, and APD_90_ were recorded after application of propofol. (a) Representative changes in APA parameters. (b) Representative changes in RPF parameters. (c) Representative changes in APD_90_ parameters. (d) Representative changes in VDD parameters. APA, amplitude of action potential; RPF, rate of pacemaker firing; APD_90_, APD at 90% repolarization; VDD, velocity of diastolic depolarization in phase 4. Data are expressed as mean ± SD. ^*∗*^*P* < 0.05 vs. control; ^#^*P* < 0.05 vs. 1 *µ*M propofol; ^+^*P* < 0.05 vs. 3 *µ*M propofol.

**Figure 3:** Electrophysiological effects of propofol on sinoatrial node pacemaker cells. (a) Control. (b) 1 *µ*M propofol. (c) 3 *µ*M propofol. (d) 5 *µ*M propofol. (e) 10 *µ*M propofol.

**Table 1:** Effect of propofol on heart rate in rabbits (beats/min).

Group	T0	T1	T2	T3	T4	T5
C	276 ± 65	274 ± 57	282 ± 48	285 ± 60	275 ± 63	280 ± 52
P1	278 ± 54	257 ± 49^*∗*^	240 ± 43^*∗*^	218 ± 42^*∗*^	210 ± 61^*∗*^	275 ± 53
P2	275 ± 68	250 ± 62^*∗*^	228 ± 41^*∗*^^#^	200 ± 59^*∗*^^#^	192 ± 57^*∗*^^#^	270 ± 46
P3	280 ± 44	240 ± 61^*∗*^^#^	211 ± 56^*∗*^^#+^	193 ± 64^*∗*^^#+^	175 ± 61^*∗*^^#+^	272 ± 73

*n* = 6. ^*∗*^*P* < 0.05 vs. sham; ^#^*P* < 0.05 vs. P1; ^+^*P* < 0.05 vs. P2. C: sham group; P1: 5 mg/kg propofol group; P2: 10 mg/kg propofol group; P3: 15 mg/kg propofol group.

**Table 2:** Effect of propofol on the discharge frequency of vagus nerve in rabbits (Hz).

Group	T0	T1	T2	T3	T4	T5
C	644 ± 27	640 ± 32	638 ± 29	642 ± 24	644 ± 31	638 ± 38
P1	645 ± 14	685 ± 36^*∗*^	700 ± 46^*∗*^	711 ± 40^*∗*^	722 ± 35^*∗*^	646 ± 30
P2	642 ± 19	694 ± 22^*∗*^	719 ± 34^*∗*^^#^	729 ± 21^*∗*^^#^	740 ± 19^*∗*^^#^	640 ± 23
P3	639 ± 17	703 ± 18^*∗*^^#^	734 ± 33^*∗*^^#+^	745 ± 27^*∗*^^#+^	752 ± 31^*∗*^^#+^	637 ± 28

*n* = 6. ^*∗*^*P* < 0.05 vs. sham; ^#^*P* < 0.05 vs. P1; ^+^*P* < 0.05 vs. P2. C: sham group; P1: 5 mg/kg propofol group; P2: 10 mg/kg propofol group; P3: 15 mg/kg propofol group.

**Table 3:** Effects of propofol on action potentials in rabbit sinoatrial node pacemaker cells.

Concentration	APA (mV)	VDD (mV/s)	RPF (beats/min)	APD_90_ (ms)
Control	74.5 ± 6.3	65.8 ± 3.9	125.3 ± 10.7	134.8 ± 7.7
1* µ*M	67.6 ± 7.7	55.6 ± 4.3^*∗*^	115.0 ± 12.9	140.2 ± 7.1
3 *µ*M	60.1 ± 5.1^*∗*^^#^	43.6 ± 6.7^*∗*^^#^	108.3 ± 12.4^*∗*^	149.4 ± 6.3^*∗*^
5 *µ*M	55.1 ± 6.4^*∗*^^#+^	34.5 ± 5.2^*∗*^^#+^	99.5 ± 11.8^*∗*^^#^	156.1 ± 9.0^*∗*^^#+^
10 *µ*M	53.4 ± 5.3^*∗*^^#+^	33.4 ± 6.0^*∗*^^#+^	98.2 ± 10.2^*∗*^^#+^	158.6 ± 8.8^*∗*^^#+^

*n* = 6. ^*∗*^*P* < 0.05 vs. control; ^#^*P* < 0.05 vs. 1 *µ*M propofol; ^+^*P* < 0.05 vs. 3 *µ*M propofol. APA, amplitude of action potential; RPF, rate of pacemaker firing; APD_90_, APD at 90% repolarization; VDD, velocity of diastolic depolarization in phase 4.

## Data Availability

The simulation experiment data used to support the findings of this study are available from the corresponding author upon request.

## References

[1] Guerrier G., Rothschild P.-R., Bonnet C., Monnet D., Baillard C. (2019). Safety of low-dose propofol in non-fasted patients undergoing cataract surgery: a prospective cohort study. *British Journal of Anaesthesia*.

[2] Trapani G., Altomare C., Sanna E., Biggio G., Liso G. (2000). Propofol in anesthesia. Mechanism of action, structure-activity relationships, and drug delivery. *Current Medicinal Chemistry*.

[3] Tramèr M. R., Moore R. A., McQuay H. J. (1997). Propofol and bradycardia: causation, frequency and severity. *British Journal of Anaesthesia*.

[4] Hemphill S., McMenamin L., Bellamy M. C., Hopkins P. M. (2019). Propofol infusion syndrome: a structured literature review and analysis of published case reports. *British Journal of Anaesthesia*.

[5] Matsushima M., Kimura S., Kitaura A. (2021). Propofol suppresses the His‐ventricular conduction in paediatric patients. *Journal of Clinical Pharmacy and Therapeutics*.

[6] Kanaya N., Hirata N., Kurosawa S., Nakayama M., Namiki A. (2003). Differential effects of propofol and sevoflurane on heart rate variability. *Anesthesiology*.

[7] Hausburg M. A., Banton K. L., Roman P. E. (2020). Effects of propofol on ischemia-reperfusion and traumatic brain injury. *Journal of Critical Care*.

[8] He M., Sun H., Pang J. (2018). Propofol alleviates hypoxia-induced nerve injury in PC-12 cells by up-regulation of microRNA-153. *BMC Anesthesiology*.

[9] Sahinovic M. M., Struys M. M. R. F., Absalom A. R. (2018). Clinical pharmacokinetics and pharmacodynamics of propofol. *Clinical Pharmacokinetics*.

[10] Marik P. (2004). Propofol: therapeutic indications and side-effects. *Current Pharmaceutical Design*.

[11] Saeki T., Nishimura M., Sato N., Fujinami T., Watanabe Y. (1995). Electrophysiological demonstration and activation of *μ*-opioid receptors in the rabbit sinoatrial node. *Journal of Cardiovascular Pharmacology*.

[12] Liu Z., Zhang J., Zhang F., Chang Y. (2020). Propofol post-conditioning lessens renal ischemia/reperfusion-induced acute lung injury associated with autophagy and apoptosis through MAPK signals in rats. *Gene*.

[13] Zhang L., Ruan Z., Liang J. (2018). Protective effect of propofol on ischemia-reperfusion injury detected by HPLC-MS/MS targeted metabolic profiling. *European Journal of Pharmacology*.

